The article "Blood Pressure Model Based on Hybrid Feature Convolution Neural Network in Promoting Rehabilitation of Patients with Hypertensive Intracerebral Hemorrhage" was published in 2021. Journal: Comput Math Methods Med.

# Blood Pressure Model Based on Hybrid Feature Convolution Neural Network in Promoting Rehabilitation of Patients with Hypertensive Intracerebral Hemorrhage

**DOI:** 10.1155/2021/1980408

**Published:** 2021-12-07

**Authors:** Zhixia Zheng, Limei Bai, Shaoquan Li

**Affiliations:** Department of Neurosurgery, Cangzhou Central Hospital, Hebei 061001, China

## Abstract

**Objective:**

Accurate prediction of the rise of blood pressure is essential for the hypertensive intracerebral hemorrhage. This study uses the hybrid feature convolution neural network to establish the blood pressure model instead of the traditional method of pulse waves.

**Methods:**

The pulse waves of 100 patients were collected, and the pulse wave was decomposed into three bell wave compound forms to obtain the accurate pulse wave propagation time. Then, the mixed feature convolution neural network model ABP-net was proposed, which combined the pulse wave propagation time characteristics with the pulse wave waveform characteristics automatically extracted by one-dimensional convolution to predict the arterial blood pressure. Finally, according to the prediction results, 20 patients were treated before the high blood pressure appeared (model group), and another 20 patients with a daily fixed treatment scheme were selected as the control group.

**Results:**

In 80 training sets, compared with linear regression and the random forest method, the hybrid feature convolution neural network has higher accuracy in predicting blood pressure. In 20 test sets, the blood pressure error was eliminated within 5 mmHg. The total effective rate in the model group and the control group was 95.0% and 85.0%, respectively (*P* = 0.035). After treatment, the scores of self-care ability of daily life and limb motor function in the model group were higher than those in the control group (*P* < 0.05). There were 8 cases (13.6%) in the model group and 17 cases (28.3%) in the control group due to the recurrence of cerebrovascular accident (*P* = 0.043).

**Conclusion:**

Drug treatment guided by a blood pressure model based on a hybrid feature convolution neural network for patients with hypertensive cerebral hemorrhage can significantly and smoothly reduce blood pressure, promote the health recovery, and reduce the occurrence of cerebrovascular accidents.

## 1. Introduction

Hypertensive intracerebral hemorrhage is a typical cerebrovascular emergency and critical disease in neurosurgery [1]. It is often seen in middle-aged and older people. Patients with high blood pressure have a one-third chance of developing cerebral hemorrhage, while about 95% of patients with cerebral hemorrhage suffer from hypertension [2]. The disease is acute, rapid, and dangerous and has high morbidity and mortality. According to the literature, the early mortality rate can be as high as 49.4%, and less than half of the survivors can live [3]. Surgical treatment has always been an important treatment for hypertensive intracerebral hemorrhage [4].

However, multiple causes may induce readmission in the postoperative recovery period. The disability and mortality rates are significantly higher than those of the first bleeding, and the prognosis is lacking [5]. Rebleeding is a common cause for readmission, and it is related to many risk factors, especially the control of blood pressure [6]. Blood pressure is affected by many factors and changes in real time, so continuous blood pressure monitoring is essential for doctors to diagnose and control patients' conditions.

In recent years, medical research has shown that cerebrovascular events' timing is closely related to the circadian rhythm of human blood pressure [7]. With the birth and development of time medicine and its penetration and promotion of nursing discipline, today's nursing model has been derived, and time nursing has begun to attract scholars' attention [8–12]. So far, many kinds of regression models have been established for continuous measurement of blood pressure, among which pulse wave velocity (PWV) is the most common. PWV is the propagation velocity of the pressure wave in blood vessels. It is often estimated by the pulse transit time (PTT), which is the time when the heart beats around the body. There was a significant correlation between blood pressure and PTT. However, the accuracy of different PTT regression models for predicting blood pressure was low.

Machine learning has made great progress in the establishment of various prediction models [13, 14]. To solve the above problems, we first propose a pulse wave decomposition algorithm to locate the repetitive pulse wave location and obtain the accurate PTT. Then, a new blood pressure prediction model is proposed, which is a hybrid feature convolution neural network. Based on the traditional fully connected neural network constructed by PTT, the pulse wave features extracted automatically are added to predict blood pressure; then, the blood pressure model is established. Finally, we also use the model to guide the treatment of hypertensive intracerebral hemorrhage.

## 2. Materials and Methods

### 2.1. General Materials

A total of 120 patients with hypertensive intracerebral hemorrhage who were hospitalized in our hospital were selected. There were 74 males and 46 females, aged 56 ± 14 years old. The selection criteria were as follows: (1) patients had hypertensive cerebral hemorrhage diagnosed by computed tomography (CT) after admission and confirmed by operation; (2) patients were admitted to the hospital within 3 h after the onset of the disease, craniocerebral surgery was performed within 24 h after the onset of the disease, and the postoperative blood pressure of the patients was above 165/95 mmHg; (3) mental retardation was excluded; and (4) other chronic diseases were excluded.

The vital sign signals collected from the medical information system in 80 patients were used as the training sets. The remaining 40 patients were used as the testing sets and were randomly divided into two groups. The established model is verified in 20 patients, and they were treated before the high blood pressure appeared (model group), and another 20 patients with a daily fixed treatment scheme were selected as the control group. There was no significant difference in gender, education level, and course of disease between the two groups.

### 2.2. Blood Pressure Modeling Method Based on Hybrid Feature Convolution Neural Network

The algorithm flowchart of this study is shown in Figure 1.

#### 2.2.1. Data Acquisition and Preprocessing

The signals used in this study include the electrocardiogram (ECG), photoplethysmograph (PPG), and arterial blood pressure (ABP). PPG is the finger volume pulse wave. The pretreatment includes the following stages:

1. *Remove baseline drift*: wavelet decomposition is used to remove the low frequency ECG and PPG parts to achieve the purpose of removing the baseline
2. *Division of cardiac cycle*: firstly, the R wave peak of the ECG is chosen as the starting point of the cardiac cycle; secondly, the cardiac cycle of PPG and ABP was divided. According to the time relationship, the first cardiac cycle of PPG and ABP was found from each R wave peak, and the ECG starting point and PPG and ABP segments belonging to the same cardiac cycle were combined; finally, the true systolic blood pressure (SBP) and diastolic blood pressure (DBP) were determined according to the ABP fragment
3. *Noise sample removal*: rules are used to remove the cardiac cycle with obvious abnormal waveform shape, such as the long cardiac cycle caused by the wrong division of the starting point in PPG and ABP and the distortion of signal shape caused by equipment acquisition

#### 2.2.2. PTT Feature Extraction

The pulse wave contains rich physiological information. The main characteristic points are pulse wave starting point A, main wave peak B, tide wave starting point C, tide wave ending point D, descending gorge E, and repetition wave peak F (Figure 2).

The main wave peak B is caused by ventricular contraction, blood from left ventricular to aorta, reflecting the ability of ventricular ejection and compliance of blood vessels, etc. The peak F of the heavy pulse wave is caused by the diastolic period of the heart; the closure of the aortic valve prevents blood from returning to the ventricle, reflecting the elasticity of the artery and the closing function of the active pulse valve. B and F are the two most important characteristic points in a cardiac cycle. Therefore, B and F are selected as the termination points to calculate PTT and are recorded as PTT-p and PTT-d, respectively, as shown in Figure 3.

B is obtained by calculating the maximum position of PPG in a cardiac cycle, and F is obtained by continuous wavelet decomposition of PPG with gaus1 wavelet basis. The first zero crossing point after B is E, and the second zero crossing point is F.

#### 2.2.3. Waveform Feature Extraction and Model Construction

This study proposes a new blood pressure prediction model ABP-net, which uses 1D-CNN to automatically extract the waveform features of PPG and predict blood pressure, and solves the problem of feature points being difficult to extract, as shown in Figure 4.

ABP-net is a convolutional neural network with mixed features, and the grey identification part is a model constructed with PTT features. In this study, PPG segments of the same cardiac cycle are also added to the network as input. One-dimensional convolution is used to extract the waveform features of the pulse wave, and the full connection layer is used to synthesize and select the extracted waveform features, and then, PTT features are used for blood pressure prediction. The model input contains two types of features: PTT is the traditional numerical feature and PPG is the formal feature (such as signal and image). ABP-net effectively integrates numerical features and formal features, which provides a new idea for using different types of features to model together, and improves the effectiveness and accuracy of the model by using the association between the two types of features and the output. ABP-net contains a variety of processing modules, and the dotted part is the residual structure.

The input-output feature maps in Conv-1D are all 1-dimensional; for a single sample, let *μ*_*i*_(*x*)(*i* = 1, 2, ⋯, *N*) be the *x*-th node of the *i*-th feature map at input and *N* the number of input feature maps, *v*_*j*_(*x*)(*j* = 1, 2, ⋯, *M*)  the *x*-th node of the *j*-th feature map at output and *M* the number of output feature maps, then Conv-1D is operated as follows:

(1) $$\begin{array}{c} v_{j}\left(x\right)=\overset{N}{\underset{i=1}{\sum }}\overset{K-1}{\underset{p=0}{\sum }}k_{i,j}\left(p\right)∙u_{i}\left(xS+p\right)+b_{j}, \end{array}$$

where *k*_*i*,*j*_ is the convolution kernel, connecting the two feature maps *u*_*i*_ and *v*_*j*_, the length of the convolution kernel is *K*, *S* is the sliding step of the convolution kernel, and *b*_*j*_ is the bias.

BN solves the problem that the distribution of inputs at a certain layer in a deep network changes due to previous changes in network parameters. Let a batch be *B* = {*x*_1_, *x*_2_, ⋯, *x*_*n*_}  and the algorithm be as follows:

(2) $$\begin{array}{c} u_{B}=\frac{1}{n}\overset{n}{\underset{i=1}{\sum }}x_{i}, \end{array}$$

(3) $$\begin{array}{c} \sigma_{B}^{2}=\frac{1}{n}\overset{n}{\underset{i=1}{\sum }}{\left(x_{i}-\mu_{B}\right)}^{2}, \end{array}$$

(4) $$\begin{array}{c} {\hat{x}}_{i}=\frac{x_{i}-\mu_{B}}{\sqrt{\sigma_{B}^{2}+\varepsilon }}, \end{array}$$

(5) $$\begin{array}{c} y_{i}=\gamma {\hat{x}}_{i}+\beta , \end{array}$$

where *μ*_*B*_ is the expectation of sample set *B*, *σ*_*B*_^2^ is the variance, *y*_*i*_ is the result normalized to batches of *x*_*i*_, and *γ*  and *β*  are parameters to be learned, determined by training. When used in the 1-dimensional convolution section, set *B* is the set of values over all positions of that feature map for all samples of that match on the same feature map.

The activation function enables the model to obtain nonlinear modeling capability, and the ReLU function

(6) $$\begin{array}{c} \text{f}\left(\text{x}\right)=\max\left(0,\text{x}\right), \end{array}$$

does not cause a gradient disappearance problem and is computationally simple, making the model forward computing faster.

Pooling can reduce feature dimensionality while acquiring the main information in a feature map and is divided into two types, maximum pooling and average pooling.

Pooling of maxima:

(7) $$\begin{array}{c} p_{i}\left(x\right)=\max\left\{u_{i}\left(p\right)\;|\;xS《p《xS+K-1\right\}. \end{array}$$

Pooling of means:

(8) $$\begin{array}{c} p_{i}\left(x\right)=\text{mean}\left\{u_{i}\left(p\right)\;|\;xS《p《xS+K-1\right\}. \end{array}$$

*p*_*i*_ is the result after pooling of eigenvectors *u*_*i*_, *K* is the pooling window size, and *S* is the window sliding step.

The other modules are the traditional neural network modules, FC is the fully connected layer, and AVG is the input format that is needed to convert the output of the convolutional layer into a fully connected layer with the method of averaging.

#### 2.2.4. Model Training

Model training is to update the network parameters iteratively to make the loss function converge to the global minimum in the training set. ABP-net is a regression model with blood pressure as the output. The loss function is defined as the mean square error (MSE). Let *y* = (*y*_1_, *y*_2_, ⋯, *y*_*n*_) be the real output of blood pressure and $\hat{y}=\left({\hat{y}}_{1},{\hat{y}}_{2},\cdots ,{\hat{y}}_{n}\right)$ be the model output of blood pressure

(9) $$\begin{array}{c} \text{MSE}=\frac{1}{n}\overset{n}{\underset{i=1}{\sum }}{\left(y_{i}-{\overset{\wedge }{y}}_{i}\right)}^{2}, \end{array}$$

where *n* is the size of a batch. In this study, batch gradient descent method is used to train the model and optimize the MSE.

### 2.3. Targeted Treatment

Patients in the control group received the routine blood pressure control measures: antihypertensive drugs three times a day and the rehabilitation did not control the time. The observation group used the model-predicted blood pressure increase pad to give targeted treatment. This seems to be a routine treatment after this.

According to the circadian rhythm fluctuation of blood pressure in patients with hypertensive intracerebral hemorrhage, the model group was given nursing intervention measures such as adjusting medication time and guiding patients' early limb function training according to the circadian rhythm fluctuation of blood pressure. The detailed biological clock control methods were as follows:

1. *Medication control*: the patients adopted the best medication time according to the physiological rhythm: three times per day at 6:00, 15:00, and 22:00; two times per day at 6:00 and 22:00; and one time per day at 6:00
2. *Early limb function training*: the training time of patients was based on the diurnal variation of blood pressure and avoided the peak time of blood pressure. Generally, they were selected from 6:00 to 7:00, 14:00 to 16:00, and 19:00 to 21:00. The blood pressure peak period was reduced, the activity was moderate, and the rest was increased to prevent the recurrence of cerebrovascular accident due to the further increase of blood pressure after the activity. The limb function training included passive limb movement exercise, active body movement, and daily life self-care activity training
3. *Follow-up*: strengthen follow-up supervision after discharge. Taking the family as the center, the patients can understand the harmfulness of hypertensive cerebral hemorrhage and the importance of continuous medication and limb function training, improve the medication compliance of patients, teach the sense and family members to measure blood pressure, and enhance the self-care ability of patients

### 2.4. Observation Index

Via follow-up monitoring for 1 year, the antihypertensive effect and recurrence of the cerebrovascular accident in the two groups were monitored and compared. The Barthel score was used to evaluate the ability of daily living. The Fugl-Meyer score was used to evaluate limb motor function.

The blood pressure changes at 6:00, 4:00, 18:00, and 22:00 every day were compared to determine the measurement position, time, and sphygmomanometer, and the therapeutic effect was determined by a specially assigned person as follows: (1) *markedly effective*: the systolic and diastolic blood pressure decreased to the normal level or the diastolic blood pressure decreased by 10 mmHg and fell to the normal range; (2) *effective*: the effective blood pressure decreased significantly, but did not fall to the normal range, or the diastolic blood pressure decreased less than 10 mmHg but returned to normal or the diastolic blood pressure decreased by 10-19 mmHg or the systolic blood pressure decreased more than 40 mmHg; and (3) *invalid*: the blood pressure drop did not reach the effective index.

### 2.5. Statistical Treatment

The age, Barthel score, and Fugl-Meyer score of the two groups were compared by *t* test; the gender, education level, treatment effectiveness, and readmission rate of the two groups were compared by chi square test.

## 3. Results

### 3.1. The Validity of the Model

For each model, the prediction accuracy of DBP is higher, which indicates that DBP has higher correlation with PTT and PPG. For the traditional regression model, the model constructed by PPG is better than the model constructed by PTT, but the accuracy is lower than that of the ABP-net model, which shows that the ABP-net model is effective for the integration of PTT features and PPG features and has greater advantages than other models (Table 1).

### 3.2. Antihypertensive Rate

The antihypertensive effect of the two groups is shown in Figure 5. As the total effective rate was calculated by the sum of markedly effective rate and effective rate, the total effective rate in the model group and control group was 95.0% and 85.0%, respectively, and the difference was statistically significant (*χ*^2^ = 4.444, *P* = 0.035).

### 3.3. Comparison of Daily Life Self-Care Ability and Limb Motor Function

Compared with the data before treatment, the daily life self-care ability and limb motor function after treatment in all the two groups were improved. After treatment, the score of the model group was higher than that of the control group (*P* < 0.05). The details are shown in Figure 6.

### 3.4. Readmission of Recurrent Cerebrovascular Accident

Eight (13.3%) patients in the model group and 17 (28.3%) patients in the control group were readmitted to the hospital because of recurrence of cerebrovascular accident. The recurrent rate between the two groups was statistically significant (*χ*^2^ = 4.093, *P* = 0.043).

## 4. Discussion

Hypertensive intracerebral hemorrhage is a common primary intracerebral hemorrhage, which is caused by the rupture of blood vessels when blood pressure rises abruptly on the basis of cerebral artery disease caused by hypertension. In recent years, the incidence rate has increased year by year, about 81/10^5^, and the mortality rate of cerebral hemorrhage patients is 38%~43% [15]. For patients with hypertensive intracerebral hemorrhage, we should not only grasp the best treatment time and take the best surgical treatment but also actively take effective nursing measures after operation, so as to ensure the effect of surgical treatment and reduce the incidence of complications and mortality [16]. In the recovery period of hypertensive intracerebral hemorrhage, many factors may induce rebleeding and other cerebrovascular accidents, and the risk may be reduced by active family, scientific, and effective nursing.

With the exploration of the physiological and pathological rhythm of hypertensive cerebral hemorrhage and the time rhythm of drug action, it has been recognized that the drug treatment effect of hypertensive cerebral hemorrhage is related not only to the pharmacological effect of antihypertensive drugs but also to the blood pressure fluctuation time rule, the medication time rule of patients itself [17]. With the birth and development of time medicine, time nursing has been gradually recognized by people. It refers to a new discipline wherein nurses use the intrinsic rhythm of the body itself to care for patients' psychological factors, medication time, physiology, and pathology [18]. In this study, according to the time rhythm of hypertensive intracerebral hemorrhage, we applied time nursing to comprehensive treatment and nursing intervention measures. The results showed that time nursing can effectively and steadily reduce blood pressure and reduce the occurrence of cerebrovascular accidents, so as to improve the quality of life of patients with hypertensive intracerebral hemorrhage.

The circadian rhythm curve of blood pressure in patients with hypertensive intracerebral hemorrhage is similar to that in normal people, but the overall blood pressure level is higher and the fluctuation range is larger. Even if the blood pressure has decreased after treatment, the rhythm can still exist. At 2:00-3:00 in the morning, it was at the lowest point and then showed an upward trend. After getting up in the morning, it rose rapidly, reaching the first peak at about 8:00-9:00 am and slightly higher at 5:00-6:00 p.m., which was the second peak, and then began to decline slowly. Therefore, the 24 h ambulatory blood pressure monitoring curve showed a double peak and a valley. In the traditional method of administration, the drug was administered by the method of average distribution, three time per day [19]. As the drug was not given according to the time rhythm, two adverse effects can occur. On the one hand, in some patients, the drug administration interval is too long and the blood drug concentration drops rapidly, which affects the curative effect; on the other hand, the drug accumulation is too much and causes poisoning of the drug's therapeutic effect in the human body [20].

In this study, we applied time nursing, according to the time law of circadian blood pressure changes; the patients with hypertensive intracerebral hemorrhage were given medicine three times per day at 6:00, 15:00, and 22:00; two times per day at 6:00 and 22:00; and one time per day at 6:00. The blood pressure of hypertensive cerebral hemorrhage patients increased at 6:00, and the concentration of drugs in the blood was very low after overnight metabolism. At 6:00, the effective pharmacological actions in the body can be supplemented as soon as possible, so that the peak effect of antihypertensive drugs corresponds to the morning blood pressure peak, which is conducive to the control of morning peak blood pressure. At 15:00, the antihypertensive drug is given before the second peak of the blood pressure fluctuation, which can reduce blood pressure in time and reduce the damage to target organs after the blood pressure rises. The effective blood concentration can be maintained at night by administration at 22:00 and can reduce the incidence of complications.

And then, the drug treatment under the guidance of the hybrid feature convolution neural network was used, and the blood pressure prediction model of patients with hypertensive cerebral hemorrhage was established. Using the model to predict the blood pressure increase point of patients, targeted treatment for patients can significantly and smoothly reduce blood pressure, promote health recovery, and reduce the occurrence of cerebrovascular accidents.

Early limb function training can promote the reorganization of the central nervous function, significantly improve the body motor function, reduce the degree of damage and disability, promote the recovery of nerve function, improve the quality of life, and reduce the burden of society [21]. According to the diurnal and nocturnal changes, the blood pressure peak time is generally selected as 6:00-7:00, 14:00-16:00, and 19:00-21:00. During the peak blood pressure, moderate movement and increased rest should be adopted to prevent the recurrence of cerebrovascular accident.

## 5. Conclusions

In summary, mastering the drug treatment under the guidance of a hybrid feature convolution neural network and establishing the blood pressure prediction model of patients with hypertensive intracerebral hemorrhage can reduce the blood pressure of patients with hypertensive intracerebral hemorrhage, promote health recovery, and reduce the occurrence of cerebrovascular accidents. It has very important practical significance to improve the survival quality of patients with hypertensive intracerebral hemorrhage, which is worthy of further clinical investigation.

## Figures and Tables

**Figure 1:** Algorithm flowchart of blood pressure modeling.

**Figure 2:** Single cardiac cycle pulse wave feature points.

**Figure 3:** PTT feature extraction method.

**Figure 4:** ABP-net network structure.

**Figure 5:** Antihypertensive effect in the model group (a) and control group (b).

**Figure 6:** Comparison of daily life self-care ability and limb motor function in two groups: (a) before treatment; (b) after treatment.

**Table 1:** Blood pressure model predicts SBP and DBP accuracy comparison.

Methods	SBP (mmHg)		DBP (mmHg)	
	PTT	PPG	PPT	PPG
ABP-net	3.32 ± 0.76	3.69 ± 0.92	1.77 ± 0.31	1.95 ± 0.39
Linear regression	6.52 ± 2.43	6.24 ± 1.85	3.44 ± 0.93	3.05 ± 0.69
Random forest	6.91 ± 2.31	4.51 ± 1.16	3.31 ± 0.87	2.22 ± 0.44

## Data Availability

All data analyzed during this study are available from the corresponding author upon request.
